# Augmented Reality Navigation for Stereoscopic Laparoscopic Anatomical Hepatectomy of Primary Liver Cancer: Preliminary Experience

**DOI:** 10.3389/fonc.2021.663236

**Published:** 2021-03-25

**Authors:** Weiqi Zhang, Wen Zhu, Jian Yang, Nan Xiang, Ning Zeng, Haoyu Hu, Fucang Jia, Chihua Fang

**Affiliations:** ^1^ Department of Hepatobiliary Surgery, Zhujiang Hospital, Southern Medical University, Guangzhou, China; ^2^ Guangdong Provincial Clinical and Engineering Center of Digital Medicine, Guangzhou, China; ^3^ Research Laboratory for Medical Imaging and Digital Surgery, Shenzhen Institutes of Advanced Technology, Chinese Academy of Sciences, Shenzhen, China

**Keywords:** laparoscopic surgical navigation, augmented reality, three-dimensional laparoscopy, anatomical hepatectomy, primary liver cancer

## Abstract

**Background:**

Accurate determination of intrahepatic anatomy remains challenging for laparoscopic anatomical hepatectomy (LAH). Laparoscopic augmented reality navigation (LARN) is expected to facilitate LAH of primary liver cancer (PLC) by identifying the exact location of tumors and vessels. The study was to evaluate the safety and effectiveness of our independently developed LARN system in LAH of PLC.

**Methods:**

From May 2018 to July 2020, the study included 85 PLC patients who underwent three-dimensional (3D) LAH. According to whether LARN was performed during the operation, the patients were divided into the intraoperative navigation (IN) group and the non-intraoperative navigation (NIN) group. We compared the preoperative data, perioperative results and postoperative complications between the two groups, and introduced our preliminary experience of this novel technology in LAH.

**Results:**

There were 44 and 41 PLC patients in the IN group and the NIN group, respectively. No significant differences were found in preoperative characteristics and any of the resection-related complications between the two groups (All *P* > 0.05). Compared with the NIN group, the IN group had significantly less operative bleeding (*P* = 0.002), lower delta Hb% (*P* = 0.039), lower blood transfusion rate (*P* < 0.001), and reduced postoperative hospital stay (*P* = 0.003). For the IN group, the successful fusion of simulated surgical planning and operative scene helped to determine the extent of resection.

**Conclusions:**

The LARN contributed to the identification of important anatomical structures during LAH of PLC. It reduced vascular injury and accelerated postoperative recovery, showing a potential application prospects in liver surgery.

## Introduction

Primary liver cancer (PLC) is the fourth most common cause of cancer-related death worldwide (second in males), and its incidence is steadily increasing (1). Anatomical hepatectomy (AH) is one of the surgical methods for PLC, which refers to the resection of hepatic area innervated by portal vein (PV) and its branches (2). With the development of laparoscopic technique, an increasing number of AH can be performed under laparoscopy (3–5). The advent of three-dimensional (3D) laparoscopy provides surgeons with depth perception, however, laparoscopic anatomical hepatectomy (LAH) has its own technical difficulty in determining the anatomic landmark and surgical plane due to the lack of tactile feedback, limited operating space, and poor viewing angles. To alleviate these drawbacks, laparoscopic augmented reality navigation (LARN) systems, including video-based, projection-based, and see-through AR visualization methods, have been introduced to improve information on the position of intrahepatic tumors and vessels, thereby facilitating LAH (6, 7). Nevertheless, unlike rigid surgical navigation in orthopedics and neurosurgery, the impact of pneumoperitoneum, respiration, heartbeat and surgical manipulation will change the accuracy of liver surgical navigation, making it difficult to transform LARN into clinical practice (8–10).

Recently, our team developed a 3D LARN system (6). This system, combined with preoperative 3D surgical planning, provides simple, safe and real-time image navigation for LAH. In this study, the clinical outcomes of the IN group and the NIN group were compared to explore the application value of this new image navigation technology in 3D LAH of PLC.

## Methods

### Patients

Between May 2018 and July 2020, a total of 85 consecutive PLC patients undergoing 3D LAH in the Department of Hepatobiliary Surgery, Zhujiang Hospital, Southern Medical University were enrolled in the study. Inclusion criteria: (1) age ≥ 18 years, regardless of gender; (2) PLC diagnosed by enhanced computed tomography (CT) or magnetic resonance imaging scan, and confirmed by pathological examination; (3) Child–Pugh class A or B liver function. Patients with main vascular invasion or extrahepatic metastasis were excluded from the study. In the intraoperative navigation (IN) group, PLC patients received 3D LAH using the LARN system. In the non-intraoperative navigation (NIN) group, PLC patients received 3D laparoscopic AH without assistance of the LARN system. All the operations were performed by the surgical group with more than 10 years of laparoscopic hepatic resection experience. The clinical data of the two groups were collected and analyzed, including sex, age, body mass index (BMI), history of hepatitis B, liver cirrhosis, Child-Pugh classification of liver function, preoperative α-fetoprotein (AFP), preoperative carbohydrate antigen 19-9 (CA19-9), preoperative total bilirubin (TBil), preoperative hemoglobin (Hb), preoperative albumin (ALB), preoperative blood platelet (PLT) count, tumor size, tumor number, operative details, perioperative results and recurrence patterns. The amount of intraoperative blood loss was calculated by adding the contents of suction containers to the weight of laparotomy sponges at the end of the surgery. Delta Hb% was defined as (Difference between preoperative Hb and postoperative lowest Hb/preoperative Hb)×100. Clavien-Dindo classification was used to evaluate postoperative complications (11). Liver failure was determined using the “50-50 criteria” (12).

Informed consent for clinical analysis was obtained from each patient, and the study was approved and supervised by the ethics committee of Zhujiang Hospital of Southern Medical University with the batch number of 2018-GDYK-003.

### 3D Model Reconstruction and Surgical Planning

All patients in the IN group were scanned with Philips Brilliance 64- or 256-multislice spiral CT scanner to collect four-phase CT data during plain scan phase, arterial phase, portal venous phase and delayed phase. The specific scanning parameters and methods were referenced to consensus recommendations of 3D visualization for diagnosis and management of liver diseases (13). The self-developed 3D visualization system (MI-3DVS, software copyright: No.2008SR18798) was used for 3D reconstruction, and several quality control criteria were followed: (1) Patients should be instructed to hold their breath during CT scan to avoid difficulties in image segmentation and registration between different phases; (2) quality of original CT images should meet the minimum standards of 3D visualization software; (3) 3D reconstruction should be performed by qualified personnel; (4) 3D models should be manually checked and modified by a senior surgeon and an imaging physician. According to the 3D models, the anatomy and spatial distribution of the targets, including liver, biliary tract, blood vessel, tumor were defined and delineated. Furthermore, residual liver volume calculation and stimulated hepatectomy were carried out to determine the surgical plane and extent of resection.

### Laparoscopic Augmented Reality Navigation System

As described in our previous study, the LARN system consisted of preoperative model segmentation, real-time image surface reconstruction, intraoperative registration, and intraoperative posture tracking modules (Software copyright: No. 2018SR840555) (14). LARN was implemented in C^++^ and Python using the open source toolkit on the Windows 10 operating system, and the software interface is shown in **Figure 1**. The ORB-SLAM2 method was adopted to acquire the real-time camera pose and 3D information of the organ surface (15). Intraoperative real-time surgical images were collected by 3D laparoscopic (Karl Storz, Germany) camera, and the output video signal in Line-by-line format needed to be analyzed by video parser (E-hospital 3D embedded multimedia workstation GK310, China). Epiphan AV.io HD video capture card was input into the laptop to form the effect of AR image display and realize real-time fusion navigation.

**Figure 1:** 3D LARN software interface.

The spatial transformation matrix between preoperative CT image space and intraoperative laparoscopic space was obtained by Go-ICP method to realize the registration of preoperative 3D visualization model and intraoperative video image (16). If the effect of automatic registration is not satisfactory, the system will provide manual registration function. The installation, debugging, 3D model introduction, positioning and image registration of the LARN system took an average of 10 minutes. 3D models including liver, gallbladder, tumor, hepatic artery, hepatic vein and PV were assigned brown, green, yellow, red, dark blue and sky blue, respectively. Two liver surface anatomical landmarks, the inferior vena cava fossa and the fundus of gallbladder, were selected for registration. While registering, the size alignment of the liver shape was taken into account, and the projection and fusion of the 3D model were further adjusted. LARN was not performed during liver mobilization. After dissociating ligaments, the liver would undergo morphological changes due to the effects of squeezing, flipping, lifting and pulling the liver tissue and pneumoperitoneal pressure. Therefore, when dissecting the first porta hepatis, we used the vessels of hepatic hilum (PV, hepatic artery or abdominal aorta) as the registration landmarks for real-time image navigation to understand the location relationship of vascular system.

### Statistical Analysis

All statistical analyses were performed using SPSS 25.0 (IBM Corp., Armonk, NY, USA). Continuous variables were expressed as median (Range) and compared using Mann-Whitney U test. Category data were presented as number (Percentage) and compared with the χ2 test or the Fisher exact test. *P* < 0.05 was considered as indicative of statistical significance.

## Results

### Patients Characteristics

The comparison of baseline data between the IN group and the NIN group is shown in **Table 1**. Between May 2018 and July 2020, a total of 85 PLC patients were enrolled into our study, including 34 cases of right hepatectomy, 21 cases of left hepatectomy, 13 cases of right posterior sectionectomy, 8 cases of left lateral sectionectomy, 7 cases of mesohepatectomy, and 2 cases of S5+6 segmentectomy. No significant differences were noted regarding age, sex, BMI, history of hepatitis B, Child-Pugh classification of liver function, preoperative AFP, preoperative CA19-9, preoperative TBIL, preoperative Hb, preoperative ALB, preoperative PLT, tumor size, tumor number, type of AH, extent of resection and pathological result between the two groups (All *P* > 0.05).

**Table 1:** Patient Characteristics.

Characteristics	IN group (n = 44)	NIN group (n = 41)	*P* Value
*Host factors*			
Age, year, median (range)	53 (25-74)	61 (26-78)	0.381
Sex, n (%)			0.659
Male	36 (82)	35 (85)	
Female	8 (18)	6 (15)	
BMI, kg/m^2^, median (range)	22.3 (17.4-27.2)	22.1 (15.4-29.0)	0.907
Hepatitis B, n (%)	34 (77)	25 (61)	0.103
Liver cirrhosis, n (%)	21 (48)	13 (32)	0.132
Child-Pugh classification, n (%)			0.738
Class A	40 (91)	39 (95)	
Class B	4 (9)	2 (5)	
*Preoperative laboratory tests*			
AFP, ng/mL, median (range)	10.1 (1.6-79776.0)	10.7 (1.4-166690.0)	0.076
CA19-9, U/mL, median (range)	16.6 (1.1-968.6)	27.5 (0.6-431800.0)	0.208
TBil, mg/dL, median (range)	0.8 (0.4-2.4)	0.9 (0.3-8.9)	0.208
Hb, g/L, median (range)	137 (97-170)	135 (99-185)	0.264
ALB, g/L, median (range)	37.8 (28.0-59.7)	39.5 (27.3-52.9)	0.335
PLT, 10^3^/μL, median (range)	177 (14-469)	220 (30-539)	0.418
*Tumor and surgical factors*			
Tumor size	6.0 (0.6-16.0)	7.0 (1.3-18.0)	0.779
Tumor number, n (%)			
Solitary	41 (93)	38 (93)	1.000
2-3 nodules	3 (7)	2 (5)	1.000
>3 nodules	0	1 (2)	0.482
Anatomical resection, n (%)			
Left hepatectomy (S2, S3 and S4)	10 (23)	11 (27)	0.661
Right hepatectomy (S5, S6, S7 and S8)	19 (44)	15 (36)	0.535
Left lateral sectionectomy (S2+3)	2 (4)	6 (15)	0.222
Mesohepatectomy (S4, S5 and S8)	4 (9)	3 (7)	1.000
Right posterior sectionectomy (S6+7)	7 (16)	6 (15)	0.870
S5+6 segmentectomy	2 (4)	0 (0)	0.496
Extent of resection, n (%)			0.658
Minor^a^	11 (25)	12 (29)	
Major^b^	33 (75)	29 (71)	
Pathological findings, n (%)			0.843
Hepatocellular carcinoma	38 (86)	36 (88)	
Cholangiocarcinoma	6 (14)	5 (12)	

BMI, body mass index; AFP, α-fetoprotein; CA19-9, carbohydrate antigen 19-9; Hb, hemoglobin; TBil, total bilirubin; ALB, albumin; PLT, platelet.

a Removal of less than 3 hepatic segments.

b Removal of 3 or more adjacent hepatic segments.

### Perioperative Outcomes and Recurrence Patterns

The operation time, blood loss, intraoperative blood transfusion, postoperative hospital stay, resection-related complications and recurrence patterns are described in **Table 2**. We found that the intraoperative blood loss, delta Hb% and blood transfusion rate were significantly higher in the NIN group than in the IN group (*P* = 0.002, *P* = 0.039 and *P* < 0.001, respectively). In addition, the length of postoperative hospital stay in the IN group was significantly shorter than that in the NIN group (*P* = 0.003). There was no significant difference in operative time and postoperative complications between the two groups (All *P* > 0.05). All patients recovered and discharged without liver failure or perioperative death.

**Table 2:** Perioperative Outcomes and Recurrence Patterns.

	IN group (n = 44)	NIN group (n = 41)	*P* Value
Operation time, min, median (range)	300 (90-690)	300 (90-540)	0.061
Blood loss, mL, median (range)	200 (20-400)	300 (50-1000)	**0.002**
Delta Hb%^a^, median (range)	12.1 (1.3-34.6)	14.1 (6.3-57.9)	**0.039**
Intraoperative blood transfusion, n (%)			**<0.001**
Yes	5 (10)	19 (42)	
No	39 (90)	22 (58)	
Resection-related complications, n (%)			
Total	18 (41)	19 (46)	0.614
Wound infection	0 (0)	1 (2)	0.482
Abdominal hemorrhage	0 (0)	1 (2)	0.482
Lung infection	2 (5)	3 (7)	0.935
Pleural effusion	12 (27)	12 (30)	0.838
Ascites	4 (9)	2 (5)	0.738
Liver failure	0 (0)	0 (0)	–
Clavien-Dindo classification of complications, n (%)			
Grade I or II	15 (32)	14 (33)	0.996
≥Grade III	3 (7)	5 (11)	0.634
Postoperative hospital stay, day, median (range)	8 (4-14)	10 (4-23)	**0.003**
Recurrence Patterns			
Overall recurrence, n (%)	11 (25)	16 (39)	0.165
Intrahepatic, n (%)	7 (16)	12 (29)	0.140
Extrahepatic, n (%)	1 (2)	2 (5)	0.950
Intrahepatic and extrahepatic, n (%)	3 (7)	2 (5)	1.000

a (Difference between preoperative Hb and postoperative lowest Hb/preoperative Hb)×100. Bold values indicate P < 0.05.

The median follow-up for all patients was 16 months (Range, 1–32 months). By the end of follow-up, 27 patients (32%) had developed tumor recurrence, including 11 cases (25%) in the IN group and 16 cases (39%) in the NIN group. The results of overall, intrahepatic or extrahepatic recurrence were similar between the IN and NIN groups (All *P* > 0.05).

### Right Hepatectomy

The case of right hepatectomy is shown in **Figure 2**. The upper abdomen enhanced CT indicated that the lesion was located in the right liver and was closely related to the right PV (**Figure 2A**). The 3D liver model clearly showed the location of the lesion and its anatomical relationship with the hepatic vessels (**Figure 2B**). Considering hepatocellular carcinoma (HCC), we planned to perform laparoscopic right hepatectomy. Based on simulated resection results, residual liver volume accounted for 47.1% of the total liver volume (Right liver volume = 558.15 ml) (**Figure 2C**). Intraoperatively, image fusion was performed to navigate the right hepatic artery (**Figure 2D**), the main PV and the right PV (**Figure 2E**). Under real-time image navigation, a hemi-hepatic ischemic line appeared on the surface of the liver after ligation of the right PV, and the hepatic parenchyma was incised and the right hepatic vein was carefully processed (**Figure 2F**). Postoperative pathological examination revealed HCC.

**Figure 2:** LARN-assisted right hepatectomy. **(A)**, enhanced CT indicated that the lesion was in the right liver, and it was closely related to the right PV. Iodide oil deposition was found inside the lesion. **(B)**, The 3D reconstructed model showed the relationship between the lesion and hepatic vessels. **(C)**, simulated right hepatectomy was performed, and the residual liver volume ratio was 47.1%. **(D)**, intraoperative navigation of the right hepatic artery. **(E)**, intraoperative navigation of the main PV and the right PV. **(F)**, intraoperative navigation of right hepatic vein.

### Right Posterior Sectionectomy

The case of right posterior sectionectomy is shown in **Figure 3**. 3D visualization model displayed that the lesion was located in the right posterior sector (**Figure 3A**). On the basis of simulated right posterior sectionectomy, the resected liver volume was 340.12 ml (41.33%) and the residual liver volume was 482.79 ml (58.67%) (**Figure 3B**). The hepatoduodenal ligament was dissected to isolate the main PV and the right hepatic artery (**Figures 3C, D**), and the right PV was suspended under the intraoperative image navigation (**Figure 3E**). By projecting the 3D vessel model, the right PV “fluoroscopically” traveled from the liver surface, and the right posterior PV branch was further dissected and severed (**Figures 3F, G**). According to the ischemic line, the dissection of hepatic parenchyma and the management of the hepatic veins in S6 and S7 were performed with the assistance of LARN (**Figure 3H**). Postoperative pathological examination revealed cholangiocarcinoma.

**Figure 3:** LARN-assisted right posterior sectionectomy. **(A)**, the lesion was located in the right posterior sector from 3D visualization. **(B)**, the resected liver volume was calculated to be 340.12 ml (41.33%) based on simulated hepatectomy. **(C)**, intraoperative navigation of the main PV and hepatic artery. **(D)**, intraoperative navigation of the right hepatic artery. **(E)**, the right PV was suspended under the image navigation. **(F, G)**, the right posterior PV branch was dissected and severed with the assistance of LARN. **(H)**, intraoperative navigation of the hepatic veins in S6 and S7.

### S5+6 Segmentectomy

The case of S5+6 segmentectomy is described in **Figure 4**. The abdominal contrast-enhanced CT showed a mixed density lesion in the right liver with heterogeneous enhancement (**Figure 4A**). 3D reconstruction and individualized liver segmentation demonstrated that the lesion was located in the S5 and S6 (**Figures 4B, C**), and the resected liver volume was 228.52 ml (26.57%) and the residual liver volume was 631.37 ml (73.43%) (**Figure 4C**). During the operation, the lesion was observed protruding from the liver surface. We projected the 3D models onto the liver surface to show the relationship between the lesion and PVs (**Figures 4D, E**). The right PV, the right anterior PV branch and right posterior PV branch were visualized through the fused 3D reconstructed models, and the PV branches of S5 (**Figure 4F**) and S6 (**Figure 4G**) were further separated and severed to complete the corresponding liver segment resection. Middle hepatic vein processing and the ligation of S5 hepatic vein were carried out under real-time image navigation (**Figure 4H**). Postoperative pathological examination revealed HCC.

**Figure 4:** LARN-assisted S5+6 segmentectomy. **(A)**, abdominal contrast-enhanced CT scan revealed a mixed density lesion in the right liver with heterogeneous enhancement. **(B)**, the lesion was located in the S5 and S6 from 3D visualization. **(C)**, the resected liver volume was 228.52 ml (26.57%) based on simulated hepatectomy. **(D, E)**, 3D models were projected onto the liver surface to show the relationship between the lesion and PVs. **(F)**, intraoperative navigation of the PV branch of S5. **(G)**, intraoperative navigation of the PV branch of S6. **(H)**, intraoperative navigation of middle hepatic vein.

## Discussion

Laparoscopic liver resection, which has progressed over the last 20 years, has become a feasible choice for various kinds of liver lesions owing to the development of high-tech surgical techniques and equipment (17). Due to the diversity of the lesion sites and the complicated relationship with great vessels, LAH of PLC is a high-risk procedure, and suggested to be performed by senior surgeons with adequate laparoscopic experiences (18). Overdependence on the skills of surgeons may lead to vascular injury, inaccurate tumor localization, and excessive resection of normal liver tissue. 3D visualization based on preoperative CT has been proven safe and effective for hepatic vessels classification, liver segmentation, simulated hepatectomy, and measurement of liver volume (13, 19). However, it mainly plays the role of pre-resection evaluation and cannot be fused into the surgical scene. Intraoperative visualization of preoperative image data has been a research issue of software engineers, computer scientists and clinicians to improve clinical outcomes for technically challenging LAH. AR allows a real-time updated 3D virtual model of anatomical structures beneath the tissue surface such as blood vessels, nerves, lesions, etc. to be superimposed over the real-world scenario (20). Compared with AR display modes including see-through, 3D image overlay, and projector based methods (21–23), video see-through is more natural and convenient for surgeons to operate under the laparoscopic view and becomes the main form of LARN (6). Concerning the field of laparoscopic surgery, LARN based on video see-through has been gradually promoted to nephrectomy (24), pancreatoduodenectomy (25), esophagectomy (26). Because of the particularity of abdominal environment and the complexity of hepatic vascular structure, the application of LARN in liver surgery is still facing challenges. The LARN system reported in this study achieved real-time navigation of LAH by fusing the preoperative 3D models and contributed to the precise resection of PLC.

The literature on LARN in liver surgery is scarce, mainly in the form of case reports, video reports, and small series. In 2014, Kenngott et al. (27) reported a promising method of real-time image guidance in laparoscopic liver surgery by combining AR software guidance system with intraoperative C-arm cone-beam CT. In a publication by Hallet et al. (28), 3D virtual planning and AR were demonstrated to facilitate trans-thoracic approach for resection of lesions from the liver dome. Nevertheless, the above studies did not involve LAH and surgical details. In 2017, Phutane et al. (29) described a case of laparoscopic left hepatectomy with initial control of the left hepatic vein assisted by their new AR guidance system. According to their study, they completed 8 similar LARN-guided left hepatectomies with satisfactory results, showing potential application prospect of LARN in LAH. Recently, a case series including laparoscopic hemihepatectomy and segmentectomy suggested the feasibility and the potential interest of using the AR guidance software to achieve AR with a deformable model during laparoscopic hepatectomy to locate tumors (30). It was noteworthy that the AR system supplemented the tumor location information in 2 patients which was not displayed by laparoscopic ultrasonography. Due to the small sample size and the lack of control groups, comparative researches are needed to further assess the interest and efficacy of LARN during LAH.

Our proposed LARN system achieved similar functions as the above studies, and the accuracy of our LARN system has been assessed in previous pre-clinical studies on both ex vivo and vivo porcine livers (6). Preoperatively, 3D models were reconstructed using a homogeneous and standardized 3D visualization processing (13). Through a fast registration procedure, 3D images were integrated with the current patient and surgical instrument position into a unified coordinate space. The optical tracking system was used to track the position of surgical instruments (Polaris Spectra optical tracker, Northern Digital Inc., Waterloo, Ontario, Canada). The system presented an intuitive AR navigation visualization by superimposing liver, tumor and vascular models in different colors on laparoscopic images to provide detailed information for LAH. From our experience, a notable advantage of the LARN system is that the surgeons can constantly keep track of the surgical field without the distraction during critical portions of surgical procedure, which was helpful to solve the hand-eye incongruity problem of laparoscopic operation.

Massive bleeding is the major concern in LAH. So far, the main methods used to prevent and control intraoperative hemorrhage include blocking hepatic blood flow and reducing central venous pressure. However, prolonged blockade of the porta hepatis may cause hepatic ischemia-reperfusion injury and increase the occurrence of postoperative liver failure (31). In our outcomes, intraoperative blood loss and blood transfusion rate were significantly reduced in the IN group than in the NIN group. For the patients in the IN group, LARN realized the real-time fusion of preoperative 3D reconstruction models with intraoperative surgical field, thus making the adjacent relationship between lesions and intrahepatic vascular structures more stereoscopic and visualized. At the same time, LARN predicted in advance the important vessels that were encountered in the resection plane, preventing accidental bleeding of hepatic venous system and hepatic ischemia caused by injuring PV branches. For instance, the bleeding-prone middle hepatic veins, short hepatic veins, and right hepatic vein roots were well protected during right hepatectomy under the navigation. Several studies have shown that increased intraoperative blood loss and blood transfusion decrease the overall survival and recurrence-free survival of patients with hepatocellular carcinoma treated with hepatectomy (32–34). Although there was no significant difference in postoperative recurrence between the two groups, the overall recurrence rate in the IN group was noted to be lower than that in the NIN group (25% versus 39%). The LARN system is expected to improve the long-term survival of patients with PLC undergoing LAH by reducing intraoperative bleeding and transfusion requirement.

Although there was no significant difference in resection-related complications between the two groups, the postoperative hospital stay in the IN group was significantly shorter than that in the NIN group. Previous studies have long demonstrated that excessive intraoperative blood loss and blood transfusion correlate with perioperative recovery (35, 36). We believed that the difference in postoperative hospital stay was due to the reduction of intraoperative blood loss and blood transfusion rate in LAH assisted by LARN system. In addition to the morphology of the liver, tumor, and vasculature, we also projected the preoperative scheme of LAH into the surgical scene. Through the analysis of the anatomy and variation of the hepatic vessels, the individualized liver segmentation were performed according to the topological relation of PV blood flow, and meanwhile, the volume calculation of PV branch drainage area were conducted. For all the patients in the IN group, the hepatic segment and simulated surgical plane were clearly fused with the actual operation. The successful intraoperative transformation of preoperative surgical planning improved preliminary identification of target hepatic segments.

Because the study is a retrospective case-control study with selective bias, a large sample prospective randomized controlled trial should be carried out to confirm the application value of LARN in 3D LAH. Besides, the present the LARN system is limited by a short time lag, and the preoperative 3D visualization results are not completely consistent with the liver displacement and deformation caused by pneumoperitoneum, respiration, heartbeat and surgical manipulation. It is therefore advised to combine the surgical navigation system with ultrasound in complex cases to identify the location of tumor and hepatic vessel. Soft tissue deformation and intraoperative image real-time analysis still need further research to improve the real-time and accuracy of navigation.

## Conclusions

Despite the above limitations, the LARN system helped surgeons identify important anatomical structures during LAH. The unique advantages of LARN-assisted 3D LAH of PLC in our study included decreased intraoperative bleeding, transfusion requirements and length of hospital stay. The novel image navigation technology provides a reliable technical support for laparoscopic liver resection.

## Data Availability Statement

The raw data supporting the conclusions of this article will be made available by the authors, without undue reservation.

## Ethics Statement

The studies involving human participants were reviewed and approved by the ethics committee of Zhujiang Hospital of Southern Medical University. The patients/participants provided their written informed consent to participate in this study.

## Author Contributions

WQZ, WZ, FJ and CF contributed to conception and design of the study. WQZ organized the database. WQZ and HH performed the statistical analysis. WQZ wrote the first draft of the manuscript. JY, NX and NZ wrote sections of the manuscript. All authors contributed to the article and approved the submitted version.

## Funding

This work was supported by the grants from the National Key R&D Program, China (No. 2016YFC0106500), the NSFC-GD Union Foundation, China (No. U1401254), the Major Instrument Project of National Natural Science Fund, China (No. 81627805), and National High Technology Research and Development Program of China (863 program, China) (Nos. 2006AA02Z346 and 2012AA021105).

## Conflict of Interest

The authors declare that the research was conducted in the absence of any commercial or financial relationships that could be construed as a potential conflict of interest.

## References

[1] SatrianoLLewinskaMRodriguesPBanalesJMAndersenJB. Metabolic rearrangements in primary liver cancers: cause and consequences. Nat Rev Gastroenterol Hepatol (2019) 16(12):748–66. 10.1038/s41575-019-0217-8 31666728

[2] MakuuchiMHasegawaHYamazakiS. Ultrasonically guided subsegmentectomy. Surg Gynecol Obstet (1985) 161(4):346–50.2996162

[3] XuYChenMMengXLuPWangXZhangW. Laparoscopic anatomical liver resection guided by real-time indocyanine green fluorescence imaging: experience and lessons learned from the initial series in a single center. Surg Endosc (2020) 34(10):4683–91. 10.1007/s00464-020-07691-5 32500459

[4] HommaYHondaGKurataMOmeYDoiMYamamotoJ. Pure laparoscopic right posterior sectionectomy using the caudate lobe-first approach. Surg Endosc (2019) 33(11):3851–7. 10.1007/s00464-019-06877-w 31183798

[5] BerardiGWakabayashiGIgarashiKOzakiTToyotaNTsuchiyaA. Full Laparoscopic Anatomical Segment 8 Resection for Hepatocellular Carcinoma Using the Glissonian Approach with Indocyanine Green Dye Fluorescence. Ann Surg Oncol (2019) 26(8):2577–8. 10.1245/s10434-019-07422-8 31065966

[6] LuoHYinDZhangSXiaoDHeBMengF. Augmented reality navigation for liver resection with a stereoscopic laparoscope. Comput Methods Programs Biomed (2020) 187:105099. 10.1016/j.cmpb.2019.105099 31601442

[7] TangRMaLFRongZXLiMDZengJPWangXD. Augmented reality technology for preoperative planning and intraoperative navigation during hepatobiliary surgery: A review of current methods. Hepatobiliary Pancreat Dis Int (2018) 17(2):101–12. 10.1016/j.hbpd.2018.02.002 29567047

[8] SimpsonAKinghamT. Current Evidence in Image-Guided Liver Surgery. J Gastrointest Surg (2016) 20(6):1265–9. 10.1007/s11605-016-3101-7 PMC497056826956008

[9] ZygomalasAKehagiasI. Up-to-date intraoperative computer assisted solutions for liver surgery. World J Gastrointest Surg (2019) 11(1):1–10. 10.4240/wjgs.v11.i1.1 30705734PMC6354070

[10] DilleyJWRHughes-HallettAPrattPJPucherPHCamaraMDarziAW. Perfect Registration Leads to Imperfect Performance: A Randomized Trial of Multimodal Intraoperative Image Guidance. Ann Surg (2019) 269(2):236–42. 10.1097/SLA.0000000000002793 29727330

[11] DindoDDemartinesNClavienPA. Classification of surgical complications: a new proposal with evaluation in a cohort of 6336 patients and results of a survey. Ann Surg (2004) 240(2):205–13. 10.1097/01.sla.0000133083.54934.ae PMC136012315273542

[12] BalzanSBelghitiJFargesOOgataSSauvanetADelefosseD. The “50-50 criteria” on postoperative day 5: an accurate predictor of liver failure and death after hepatectomy. Ann Surg (2005) 242(6):824–8, discussion 828-9. 10.1097/01.sla.0000189131.90876.9e PMC140989116327492

[13] FangCAnJBrunoACaiXFanJFujimotoJ. Consensus recommendations of three-dimensional visualization for diagnosis and management of liver diseases. Hepatol Int (2020) 14(4):437–53. 10.1007/s12072-020-10052-y PMC736660032638296

[14] ZhangPLuoHZhuWYangJZengNFanY. Real-time navigation for laparoscopic hepatectomy using image fusion of preoperative 3D surgical plan and intraoperative indocyanine green fluorescence imaging. Surg Endosc (2020) 34(8):3449–59. 10.1007/s00464-019-07121-1 31705286

[15] MahmoudNCollinsTHostettlerASolerLDoignonCMontielJMM. Live Tracking and Dense Reconstruction for Handheld Monocular Endoscopy. IEEE Trans Med Imag (2019) 38(1):79–89. 10.1109/TMI.2018.2856109 30010552

[16] YangJLiHCampbellDJiaY. Go-ICP: A Globally Optimal Solution to 3D ICP Point-Set Registration. IEEE Trans Pattern Anal Mach Intell (2016) 38(11):2241–54. 10.1109/TPAMI.2015.2513405 26731638

[17] SynNLKabirTKohYXTanHLWangLZChinBZ. Survival Advantage of Laparoscopic Versus Open Resection For Colorectal Liver Metastases: A Meta-analysis of Individual Patient Data From Randomized Trials and Propensity-score Matched Studies. Ann Surg (2020) 272(2):253–65. 10.1097/SLA.0000000000003672 32675538

[18] XuWLiHJiZYanWZhangYZhangX. Retroperitoneal Laparoscopic Management of Paraganglioma: A Single Institute Experience. PLoS One (2016) 11(2):e0149433. 10.1371/journal.pone.0149433 26885838PMC4757081

[19] FangCZhangPQiX. Digital and intelligent liver surgery in the new era: Prospects and dilemmas. EBioMedicine (2019) 41:693–701. 10.1016/j.ebiom.2019.02.017 30773479PMC6442371

[20] LangHHuberT. Virtual and Augmented Reality in Liver Surgery. Ann Surg (2020) 271(1):e8. 10.1097/SLA.0000000000003601 31804399

[21] GolabMRBreedonPJVloeberghsM. A wearable headset for monitoring electromyography responses within spinal surgery. Eur Spine J (2016) 25(10):3214–9. 10.1007/s00586-016-4626-x 27282890

[22] WeissCRMarkerDRFischerGSFichtingerGMachadoAJCarrinoJA. Augmented reality visualization using Image-Overlay for MR-guided interventions: system description, feasibility, and initial evaluation in a spine phantom. AJR Am J Roentgenol (2011) 196(3):W305–7. 10.2214/AJR.10.5038 21343479

[23] VolonteFPuginFBucherPSugimotoMRatibOMorelP. Augmented reality and image overlay navigation with OsiriX in laparoscopic and robotic surgery: not only a matter of fashion. J Hepatobiliary Pancreat Sci (2011) 18(4):506–9. 10.1007/s00534-011-0385-6 21487758

[24] TeberDGuvenSSimpfendorferTBaumhauerMGüvenEOYencilekF. Augmented reality: a new tool to improve surgical accuracy during laparoscopic partial nephrectomy? Preliminary in vitro and in vivo results. Eur Urol (2009) 56(2):332–8. 10.1016/j.eururo.2009.05.017 19477580

[25] OndaSOkamotoTKanehiraMSuzukiFItoRFujiokaS. Identification of inferior pancreaticoduodenal artery during pancreaticoduodenectomy using augmented reality-based navigation system. J Hepatobiliary Pancreat Sci (2014) 21(4):281–7. 10.1002/jhbp.25 23970384

[26] KenngottHGNeuhausJMuller-StichBPWolfIVetterMMeinzerHP. Development of a navigation system for minimally invasive esophagectomy. Surg Endosc (2008) 22(8):1858–65. 10.1007/s00464-007-9723-9 18157716

[27] KenngottHGWagnerMGondanMNickelFNoldenMFetzerA. Real-time image guidance in laparoscopic liver surgery: first clinical experience with a guidance system based on intraoperative CT imaging. Surg Endosc (2014) 28(3):933–40. 10.1007/s00464-013-3249-0 24178862

[28] HalletJSolerLDianaMMutterDBaumertTFHabersetzerF. Trans-thoracic minimally invasive liver resection guided by augmented reality. J Am Coll Surg (2015) 220(5):e55–60. 10.1016/j.jamcollsurg.2014.12.053 25840539

[29] PhutanePBucEPoirotKOzgurEPezetDBartoliA. Preliminary trial of augmented reality performed on a laparoscopic left hepatectomy. Surg Endosc (2018) 32(1):514–5. 10.1007/s00464-017-5733-4 28791423

[30] BertrandLRAbdallahMEspinelYCalvetLPereiraBOzgurE. A case series study of augmented reality in laparoscopic liver resection with a deformable preoperative model. Surg Endosc (2020) 34(12):5642–8. 10.1007/s00464-020-07815-x 32691206

[31] ChenHJiaW. Progress in hepatectomy for hepatocellular carcinoma and peri-operation management. Genes Dis (2020) 7(3):320–7. 10.1016/j.gendis.2020.02.001 PMC745250732884986

[32] YamamotoJKosugeTTakayamaTShimadaKYamasakiSOzakiH. Perioperative blood transfusion promotes recurrence of hepatocellular carcinoma after hepatectomy. Surgery (1994) 115(3):303–9.8128355

[33] KatzSShiaJLiauKGonenMRuoLJarnaginWR. Operative blood loss independently predicts recurrence and survival after resection of hepatocellular carcinoma. Ann Surg (2009) 249(4):617–23. 10.1097/SLA.0b013e31819ed22f 19300227

[34] HaradaNShirabeKMaedaTKayashimaHIshidaTMaeharaY. Blood transfusion is associated with recurrence of hepatocellular carcinoma after hepatectomy in Child-Pugh class A patients. World J Surg (2015) 39(4):1044–51. 10.1007/s00268-014-2891-6 25446481

[35] OtsuboT. Control of the inflow and outflow system during liver resection. J Hepatobiliary Pancreat Sci (2012) 19(1):15–8. 10.1007/s00534-011-0451-0 21971691

[36] NagaoTInoueSGotoSMizutaTOmoriYKawanoN. Hepatic resection for hepatocellular carcinoma. Clinical features and long-term prognosis. Ann Surg (1987) 205(1):33–40. 10.1097/00000658-198701000-00006 3026259PMC1492876

